The article "Deep Learning-Based CT Image Characteristics and Postoperative Anal Function Restoration for Patients with Complex Anal Fistula" was published in 2021. Journal: J Healthc Eng.

# Deep Learning-Based CT Image Characteristics and Postoperative Anal Function Restoration for Patients with Complex Anal Fistula

**DOI:** 10.1155/2021/1730158

**Published:** 2021-07-28

**Authors:** Lingling Han, Yue Chen, Weidong Cheng, He Bai, Jian Wang, Miaozhi Yu

**Affiliations:** Department of Anorectal, Xinhua Hospital, Affiliated Hospital of Dalian University, Dalian 116021, China

## Abstract

**Objective:**

This study aimed to optimize the CT images of anal fistula patients using a convolutional neural network (CNN) algorithm to investigate the anal function recovery.

**Methods:**

57 patients with complex anal fistulas admitted to our hospital from January 2020 to February 2021 were selected as research subjects. Of them, CT images of 34 cases were processed using the deep learning neural network, defined as the experimental group, and the remaining unprocessed 23 cases were in the control group. Whether to process CT images depended on the patient's own wish. The imaging results were compared with the results observed during the surgery.

**Results:**

It was found that, in the experimental group, the images were clearer, with DSC = 0.89, precision = 0.98, and recall = 0.87, indicating that the processing effects were good; that the CT imaging results in the experimental group were more consistent with those observed during the surgery, and the difference was notable (*P* < 0.05). Furthermore, the experimental group had lower RP (mmHg), AMCP (mmHg) scores, and postoperative recurrence rate, with notable differences noted (*P* < 0.05).

**Conclusion:**

CT images processed by deep learning are clearer, leading to higher accuracy of preoperative diagnosis, which is suggested in clinics.

## 1. Introduction

Anal fistula, also known as “anal leakage,” is a chronic inflammatory disease that starts with the anal gland and then invades the anal canal and other normal skin tissues around the anus [1], so it is also defined as inflammatory rectum disease (RD) [2]. The anal fistula is composed of the internal opening, the fistula, and the external opening [3]. Complex anal fistula refers to the one with 2 or more internal or external openings and fistulas [4], which will bring great inconvenience to the patient's life. Its incidence is reported to be approximately 0.01%, and the young are predominantly affected [5]. There are two main treatment methods for anal fistula: one is conservative treatment based on traditional Chinese medicine, and the other is surgical treatment [6]. Nevertheless, for complex anal fistula, it is reported that the recurrence rate is as high as 30% to 50% or even 10% patients cannot be radically cured after another operation [7]. There are many factors that affect surgical treatment. The main factor is whether the positioning of the internal mouth is accurate before surgery [8, 9], and the symptomatic degree of the surgical plan will affect the probability of recurrence and the degree of anal function retention [10, 11]. The complex anal fistula is mainly treated by the surgery, with traditional Chinese medicine used for adjuvant treatment. Therefore, imaging examination is of great significance for the treatment of the complex anal fistula [12, 13].

The commonly used imaging examination methods include CT, MRI, and B-ultrasound. However, in the examination of complex anal fistulas, CT has low resolution for soft tissues, such as pelvic tissue and anal sphincter, so the accuracy rate is only 24%∼60% [14]. With the rapid development of the technology, deep learning artificial intelligence technology is widely used in the field of imaging and the neural network system has made great progress in processing medical images, which has become a research hotspot [15]. Deep learning has solved two major problems in the medical field: one is the imbalance between the number of imaging doctors and clinical imaging data; the other is the imbalance in the level of imaging doctors and the allocation of resources [16]. Deep convolutional network models can learn image features from a large number of samples, achieving end-to-end classification and detection [17].

In this study, deep learning was used to process CT images of patients with complex anal fistula, which was expected to provide guidance for the clinical diagnosis and treatment of the disease.

## 2. Methods

### 2.1. Research Subjects

57 patients admitted to our hospital from January 2019 to February 2020 who had been diagnosed with complex anal fistula were selected as research subjects, including 35 males and 22 females, aged 18∼70, with an average age of (39.2 ± 2.1) years. All patients had the CT examination, and the CT images of 34 cases were processed using the convolutional neural network, defined as the experimental group, while the remaining unprocessed 23 cases were in the control group. Whether to process CT images depended on the patient's own wish. Clinically, all patients suffered from repeated swelling and pain around the anus, accompanied by pus discharge. The duration of the disease was 3 to 12 months, and the average duration of the disease was 7 months. Physical examination revealed purulent secretions around the anus and external opening on the skin surface. This study has been approved by the ethics committee, and the patients and their families have signed the informed consent forms. Intrarectal ultrasound, MRI, and CT examinations were conducted [18].

Patients were selected as per these inclusion criteria: (1) patients diagnosed with complex anal fistulas based on digital rectal examination, (2) the disease course lasted more than 3 months, (3) the length of the fistula was more than 3 cm (including 3 cm), (4) patients who had not undergone anal fistula surgery before, and (5) those aged between 18 and 75.

Exclusion criteria were as follows: (1) patients with the complex anal fistula caused by trauma, foreign body, infection, etc.; (2) patients accompanied by severe heart, lung, liver, and kidney dysfunction; (3) patients with cervical cancer, vaginal rectal fistula, rectal tumor, etc.; (4) patients in pregnancy and lactation; (5) patients with mental disorders; (6) patients with a history of pelvic and rectal radiotherapy; (7) patients with hematopoietic, endocrine, and immune system diseases.

### 2.2. Research Methods

#### 2.2.1. CT Examination

The anti-infection treatment was performed on all patients 1 to 2 weeks before the CT scan, to improve the symptoms of the patients to meet the examination standards. 2 hours before the scan, intestine cleaning was needed. The specific process is shown in Figure 1. All patients shared an instrument and the same skilled and experienced imaging doctor who was responsible for the CT examination and image reconstruction. After image reconstruction, 2 experienced radiologists and anorectal doctors read the films together and recorded the various conditions of the fistula. Surgical plans were formulated based on the results of the CT examination and other auxiliary examinations.

#### 2.2.2. CT Image Optimization Model Based on Convolutional Neural Network Algorithm

In this research, the convolutional neural network was used to optimize CT images. The convolutional neural network consists of the convolutional layer, the pooling layer, the fully connected layer, and the deconvolutional layer [19].

First, it is needed to collect the feature map of the CT image, provided that the convolutional layer has q layers, and then the feature map of the CT image input at the q-1 layer can be expressed by equation (1). Then, the feature map of the CT image input at the *q* − 1 layer can be expressed by the following equation:

(1) $$\begin{array}{c} W\left(q,p\right)=\sum_{b=1}^{B}Y^{\left(q,p,b\right)}⊗Z^{\left(q-1,b\right)}+l^{\left(q,p\right)}, \end{array}$$

where *Y*^(*q*, *p*, *b*)^ is the convolutional kernel, *b* is the number of feature maps, and *Y*^(*q*, *p*, *b*)^ is the bias.

The activation function is a sigmoid transfer function, with a domain of (−∞, +∞) and a value domain of (0, 1). It is continuously derivable in the domain, and its reciprocal *f*'(*x*) is easy to calculate. The specific equation is as follows:

(2) $$\begin{array}{c} Y=f\left(x\right)=\frac{1}{1+e^{-x}},\\ f^{\prime }\left(x\right)=f\left(x\right)\left(1-f\left(x\right)\right). \end{array}$$

Assume *T* is the CT image and *U* represents all pixels in *T*. The segmentation part of *T* is represented by *O*. Then, the probability that *U*_*n*_ outputs *O*_*i*_ in the *i*-th path can be expressed as follows:

(3) $$\begin{array}{c} T\left(u_{n}=O_{i}\right)=\frac{1}{A}\text{exp}\left(\alpha \left(O_{i}\right)\right), \end{array}$$

where *α*(*O*_*i*_) is the value of Oi and A is a regularization term. Then, the *S*_*n*_ predicted by *U*_*n*_ can be expressed as follows:

(4) $$\begin{array}{c} Sn=argmax\left[T\left(u_{n}=O_{i}\right)\right]. \end{array}$$

The corresponding loss function is as follows:

(5) $$\begin{array}{c} L=-\frac{1}{c\;d}\sum_{n}\sum_{j}y_{nj}\text{ln}\left[T\left(u_{n}=O_{i}\right)\right]. \end{array}$$

To minimize the loss function, the stochastic gradient descent [20] is used to solve equation (5).

If the function to be fitted is expressed as follows:

(6) $$\begin{array}{c} g\left(\delta \right)=\sum_{j=0}^{l}\delta_{j}x_{j}, \end{array}$$

then the square loss function is

(7) $$\begin{array}{c} B\left(\delta \right)=\frac{1}{2m}{\sum_{i=1}^{1}\left(y^{i}-g_{\delta }\left(x^{i}\right)\right)}^{2}. \end{array}$$

The stochastic gradient descent method is used to update *δ*_*j*_ according to the sample:

(8) $$\begin{array}{c} \delta_{j}^{\prime }=\delta_{j}+\left(y^{i}-g_{\delta }\left(x^{i}\right)\right)x^{i}. \end{array}$$

The network parameters are obtained by solving equation (9), so as to obtain the network model as follows:

(9) $$\begin{array}{c} NLL\left(\delta ,M\right)=-\sum_{i=0}^{\left|M\right|}logK\left(Y=y^{\left(i\right)}|x^{\left(i\right)},\delta \right). \end{array}$$

The processed pelvic CT image through the CNN algorithm is shown in Figure 2.

### 2.3. Evaluation of the Processed CT Image

#### 2.3.1. Dice Similarity Coefficient

Dice similarity coefficient (DSC) is used to measure the similarity of two sets. The data pile can be regarded as a set, and the Dice distance is used to measure the similarity of strings.

The DSC is expressed as follows:

(10) $$\begin{array}{c} \text{DSC}=\frac{2\times \left|G\cap J\right|}{\left|G\right|+\left|J\right|}\times 100\%, \end{array}$$

where *G* is the algorithm segmentation result and *J* is the gold standard. If the DSC is closer to 1, the segmentation result is more accurate. If the DSC value is infinitely close to 0, it indicates that the segmentation result basically does not overlap with the gold standard and the segmentation fails.

#### 2.3.2. Precision

Precision refers to the proportion of the number of correctly classified positive samples to the total number of classified positive samples. A closer precision value to 1 indicates a lower error rate. The precision is expressed as follows:

(11) $$\begin{array}{c} Pre=\frac{TP}{TP+FP}\times 100\%, \end{array}$$

where TP stands for true positive, which is consistent with the gold standard; on the contrary, FP stands for false positive, which is inconsistent with the gold standard.

#### 2.3.3. Recall Rate

Recall represents the ratio of the number of correctly classified positive samples to the total number of positive samples. A closer recall value to 1 indicates an error rate that the positive samples are incorrectly classified as negative samples. Recall is expressed as follows:

(12) $$\begin{array}{c} \text{RE}=\frac{\text{TP}}{\text{TP}+\text{FN}}\times 100\%, \end{array}$$

where TP stands for true positive, FN stands for false negative, and the classification is also inconsistent with the gold standard.

Finally, it is concluded that DSC = 0.89, precision = 0.98, and recall = 0.87, which proves the feasibility of the model established in Section 2.3 and the effectiveness of image processing.

### 2.4. Observation Indicators

1. The number and position of the internal and external openings of the fistula, whether the rectum, anal sphincter, and levator ani, are associated with the fistula, the area and length of the fistula, the diameter of the fistula, the fistula trend, whether there are complicated branches, and whether there is abscess formation.
2. The recovery of anal function of the two groups of patients after surgical treatment was observed based on the CT images before and after the treatment. The Wexner anal incontinence score (Table 1) and anorectal manometry were used to evaluate its function. The parameters of anorectal manometry were anal rest pressure (ARP) and anal maximal construction pressure (AMCP).

### 2.5. Statistics

SPSS 22.0 was used to process data. Count data were expressed by percentage (%), the *Y*2 test was performed, and the rank sum test was performed for grade count data. The measurement data were expressed by the mean ± standard deviation, and the *t*-test was performed. *P* < 0.05 was the threshold for significance.

## 3. Results

### 3.1. Basic Information of Patients

As shown in Table 2, there was no notable difference in age, gender, and disease course of patients in the control group and the experimental group (*P* > 0.05), suggesting the feasibility of this study.

### 3.2. Examination Results and the Results after Surgical Treatment

After analyses, there was no difference in the external opening, while parameters such as the internal openings, the trend of the fistula, whether there was branch, whether the fistula was associated with the perianal muscle, and fistula diameter ≥ 2 mm were different from the results observed during the surgical treatment in both the experimental group and the control group, and notable differences were noted between the CT examination results and the postoperative results in both groups (*P* < 0.05), suggesting that the accuracy of CT examination was insufficient (Table 3).  Figure 3 shows the CT images of the two groups of patients. Obviously, the optimized CT images were clearer.

### 3.3. Consistency between Examination Results and Postoperative Results

Table 4 shows the consistency between the examination results and the postoperative results. It was observed that in the experimental group, the consistency of the CT examination results and the postoperative results were higher than in the control group (*P* < 0.05) (Figure 4).

### 3.4. Postoperative Anal Function Recovery and Postoperative Recurrence Rate

Table 5 shows the statistics of Wexner anal incontinence score and anorectal manometry scores. It was found that the postoperative Wexner anal incontinence score of the experimental group was lower than that of the control group, showing notable differences. Additionally, the experimental group had lower RP (mmHg), AMCP (mmHg) scores, and the postoperative recurrence rate, and the difference was notable (*P* < 0.05).  Figure 5 shows the CT images and the postoperative recovery of the two groups of patients, suggesting that both had good curative effects.

## 4. Discussion

Recently, CT imaging has been widely used in the examination of anal fistula diseases and it has certain advantages compared with other imaging techniques. Researchers have conducted a comparative study on the ordinary X-ray and CT imaging. The study found that the diagnosis of anal fistula with CT imaging is almost the same as the results of the surgery, with 96.7% of patients radically cured at one time, while the one-time cure rate of X-ray angiography is 70% [21]. The trend of fistulas is diverse and extremely irregular. Conventional two-dimensional CT images cannot fully display its distribution, and it is impossible to make accurate judgment. Hence, it is urgent to optimize the technology. There is abundant research combining CT imaging technology with three-dimensional reconstruction and applying them to the examination of anal fistulas. The results found that the accuracy, sensitivity, and specificity of the diagnosis of the internal opening of anal fistula have reached more than 90%, suggesting good effects [15]. The artificial intelligence in deep learning has made good progress in the field of medicine, especially in the field of medical imaging. Higaki et al. [22] applied fully convolutional neural networks and dense 3D conditional random field (CRF) technology to CT images for liver segmentation studies, to understand liver lesions. Tao et al. [23] applied FCN technology to the automatic analysis of cardiac magnetic resonance (CMR). In this study, the deep neural network was used to process the CT images of patients with anal fistulas. It was found that the deep learning-based CT imaging demonstrated good examination, diagnosis, and treatment results. Studies have also shown that higher accuracy of the preoperative diagnosis leads to better surgical effects, a greater possibility of recovery of anal function, and a lower probability of recurrence. Some experts have statistically studied 17 patients with complex anal fistula who underwent MSCT angiography diagnosis before the surgery. Some experts have statistically studied 17 patients with complex anal fistula who underwent multislice CT (MSCT) angiography diagnosis before the surgery. It was found that the consistency between the preoperative diagnosis and the surgical findings was close to 100%, and in the 1-year follow-up survey, there was no recurrence and the anal function recovered well [24]. In conclusion, deep learning-based CT imaging is worthy of promotion for the preoperative diagnosis of patients with anal fistula.

## 5. Conclusion

In this study, the deep learning neural network was used to process the CT images of patients with anal fistula and the preoperative imaging results were compared with the results observed during the surgery. It was found that in the experimental group, the CT imaging results were more consistent with those observed during the surgery (*P* < 0.05) and the images were clearer. Furthermore, the anal function recovery in the experimental was better.

To sum up, CT images processed by deep learning are clearer, leading to higher accuracy of preoperative diagnosis, better surgical effects, a higher possibility of recovery, and a lower recurrence rate, which is suggested in clinics.

## Figures and Tables

**Figure 1:** The specific process of CT examination.

**Figure 2:** The processed pelvic CT image.

**Figure 3:** Comparison of CT images of the two groups of patients. (a) Control group. (b) Experimental group.

**Figure 4:** Comparison of the consistency with the results observed during the surgery. (a) 2/2 or more internal openings; (b) Fistula trend; (c) Whether there are branches beside the fistula; (d) Whether it is associated with perianal muscles; (e) Diameter of fistula  ≥ 3 mm.

**Figure 5:** CT images and postoperative results. (a) CT image of the experimental group; (b) postoperative performance of the experimental group; (c) CT image of the control group; (d) postoperative performance of the control group.

**Table 1:** Wexner anal incontinence score sheet.

Grade	Characteristics
Grade *A*	The anus function is normal, and the solid, liquid, and gas are well controlled
Grade *B*	The solid and liquid is well controlled but the gas is out of control
Grade *C*	Good control of solids, but there is a little liquid, infiltrating clothing
Grade *D*	Unable to control the liquid, it will often stain the clothes
Grade *E*	Both solids and liquids are out of control

*Note.* Grades *A*, *B*, and *C* indicate good anal function, while grades *D* and *E* indicate poor anal function.

**Table 2:** The basic information of patients.

Group	Gender		Age (year)	Disease course (month)
	Male (*n* = 35)	Female (*n* = 22)		
Control group (*n* = 23)	17	10	36.8 ± 4.1	8.3 ± 3.7
Experimental group (*n* = 34)	18	12	38.2 ± 5.0	7.6 ± 4.2

**Table 3:** Comparison of examination results and postoperative results.

Anal fistula situation					
		Experimental group and postoperative results		Control group and postoperative results	
Grouping (*n* = 34)		Experimental group	Postoperative results	Control group	Postoperative results
2/2 or more internal openings		23	27	14	20
2/2 or more external openings		24	24	21	21

Fistula trend	“*Y*” sinus	12	14	7	10
	“*U*” sinus	11	15	5	8
	Other irregular sinuses	11	5	11	5

Whether there are branches beside the fistula		2	7	0	7

Whether it is associated with perianal muscles		14	17	12	19

Diameter of fistula ≥ 2 mm		24	29	13	21

**Table 4:** Consistency between the examination results and the postoperative results (*n*%).

Anal fistula situation					
Grouping		Experimental group (*n* = 34)		Control group (*n* = 23)	
2/2 or more internal openings		85.1		70.0	

Fistula trend	“*Y*” sinus	85.7	79.5	70.0	66.3
	“*U*” sinus	73.3		62.5	
Whether there are branches beside the fistula		28.6		0	
Whether it is associated with perianal muscles		82.4		61.2	
Diameter of fistula ≥ 3 mm		82.8		62.0	

**Table 5:** Postoperative anal function recovery and recurrence rate.

Grouping	Wexner anal incontinence score		Anorectal manometry		Recurrence rate (*n*%)
	Preoperative	Postoperative	ARP (mmHg)	AMCP (mmHg)	
Experimental group	0.10 ± 0.24	1.06 ± 1.34	43.43 ± 9.41	122.71 ± 12.56	20
Control group	0.14 ± 0.29	0.34 ± 0.61	47.98 ± 10.21	137.63 ± 16.99	54

## Data Availability

No data were used to support this study.
